The article "Enriched Environment Prevents Hypobaric Hypoxia Induced Memory Impairment and Neurodegeneration: Role of BDNF/PI3K/GSK3β Pathway Coupled with CREB Activation" was retracted in 2025. Reasons: duplicated images; duplicated data; duplicate publication; original data or images not available.

# Enriched Environment Prevents Hypobaric Hypoxia Induced Memory Impairment and Neurodegeneration: Role of BDNF/PI3K/GSK3β Pathway Coupled with CREB Activation

**DOI:** 10.1371/journal.pone.0062235

**Published:** 2013-05-21

**Authors:** Vishal Jain, Iswar Baitharu, Dipti Prasad, Govindasamy Ilavazhagan

**Affiliations:** 1 Department of Neurobiology, Defence Institute of Physiology and Allied Sciences (DIPAS), Delhi, India; 2 Department of Research, Hindustan University, Chennai, India; Indian Institute of Toxicology Research, India

## Abstract

Adverse environmental conditions such as hypobaric hypoxia (HH) cause memory impairment by affecting cellular machinery leading to neurodegeneration. Providing enriched environment (EE) is found to be beneficial for curing several neurodegenerative disorders. The protective role of EE in preventing HH induced neuronal death has been reported previously but the involved mechanism is still not clearly understood. The present study is an attempt to verify the impact of EE on spatial memory during HH and also to explore the possible role of neurotrophin in EE mediated neuroprotection. Signaling mechanism involved in neuroprotection was also explored. Male Sprague Dawley rats were simulated to HH condition in an Animal Decompression Chamber at an altitude of 25000 feet in standard and enriched cages for 7 days. Spatial memory was assessed through Morris Water Maze. Role of different neurotrophins was explored by gene silencing and inhibitors for their respective receptors. Further, using different blockers signaling pathway was also explored. Finding of the present study suggested that EE prevents HH mediated memory impairment and neurodegeneration. Also brain-derived neurotrophic factor (BDNF) plays a major role in EE mediated neuroprotection and it effectively prevented neurodegeneration by activating PI3K/AKT pathway resulting in GSK3β inactivation which further inhibits apoptosis. Moreover GSK3β phosphorylation and hence its inactivation upregulates CREB phosphorylation which may also accounts for activation of survival machinery in cells and provides neuroprotection. From these observations it can be postulated that EE has a therapeutic potential in amelioration of HH induced memory impairment and neurodegeneration. Hence it may be used as a non invasive and non pharmacological intervention against various neurological disorders.

## Introduction

Hypobaric hypoxia (HH) is a good model to study the pathophysiology of people staying at high altitude (HA). At HA there is low availability of oxygen due to its reduced partial pressure. It has deleterious effect on brain functions as it leads to memory impairment and cognitive dysfunctions [1]–[2]. Altered neurotransmitter synthesis, uptake and release, free radical generation and changes in gene expression and protein functions are characteristically associated with HH [3], leading to cell death and eventually memory impairment. Recent findings pointed out that severe hypoxia exposure can cause increased cellular oxidative stress with consequent damage to lipids, proteins and DNA [4]. However antioxidant supplementation showed limited neuroprotection in hypoxic and ischemic conditions which indicates involvement of other complex mechanisms that might lead to triggering of survival machinery of the cell [5].

Environmental enrichment refers to housing conditions, either home cages or exploratory chamber that facilitate enhanced sensory, cognitive and motor stimulation relative to standard housing conditions. It has been well documented that environment enrichment increases dendritic branching and length, the number of dendritic spines and the size of synapses on some neuronal populations [6]–[9]. At the behavioral level, enrichment enhances learning and memory [10]–[12], reduces memory decline in aged animals, decreases anxiety and increases exploratory activity [13]. These changes caused by enriched environment (EE) may be underlying mechanism providing neuroprotection against diverse neurological disorders.

Regarding the cellular and molecular pathways related to neuroprotection, it is reported that EE enhances the level of neurotrophin, especially brain-derived neurotrophic factor (BDNF) [14], a possible modulator of neuronal survival and plasticity [15]. Almli et al, verified that intracerebroventricular BDNF pretreatment resulted in significant protection against both Hypoxia-ischemia (HI) induced histological injury and spatial memory impairments [16]. A beneficial effect of housing in an EE on recovery from physical damage like lesion is a common finding but does EE housing prevent damage from psycho-physiological stress like HH is still a grey area.

Extracellular signal-regulated kinase (ERK) and Phsophoinositide 3 Kinase (PI3K) pathways are two main signal transduction pathways reported to play a role in BDNF-induced neuroprotection [17]. There are studies which showed that BDNF supported neuronal survival that is mediated via the ERK pathway [18] while others provide evidence of involvement of PI3K pathway [19]–[21]. A few studies also demonstrate that the p38 MAPK pathway plays a role in neuroprotection [22]–[23]. Therefore, it appears that growth factor-mediated protection to neurons varies with factors such as cell types, environmental conditions and cellular stimuli.

Our previous study showed that enriched environment provides neuroprotection against hypobaric hypoxia but fails to ameliorate oxidative stress [24]. Based on this, the present study was designed to assess the effect of EE on hypobaric hypoxia induced memory impairment and to explore the possible mechanism involved in EE mediated neuroprotection. The finding may lead to the identification of key mediators of molecular pathways which are involved in EE mediated neuroprotection against HH induced memory impairment and neurodegeneration.

## Materials and Methods

### Ethic Statement

All the experimental protocol and animal care was approved by the ethical committee of the Defence Institute of Physiology and Allied Sciences (27/1999/CPCSEA) in accordance with the guidelines of “Committee for the Purpose of Control and Supervision of Experiments on Animals” of Govt. of India. All surgery was performed under sodium pentobarbital anesthesia and all efforts were made to minimize the suffering to the animals.

### Animals

Three month old male Sprague Dawley rats (230 g) were used in the present study which were procured from animal house facility of the Institute. They were maintained in a temperature controlled room (25±2°C at 65±5% humidity) on a 12/12 h light/dark cycle with food and water available *ad libitum*. Rats were tested for anxiety levels in a plus maze and categorized into anxious and normal individuals based on their preference for closed and open arms. The normal individuals were then taken for further experimental purpose. Rats (n = 200) were divided into different experimental groups (Table 1) for further investigation.

**Table 1:** Shows experimental design describing groups, number of individuals, exposure duration and interventions.

Groups	No. of Animals (n)	Hypobaric hypoxia exposure	Standard Cage(SC)/Enriched Cage (EC)	Antagonist/Antisense
I	36	Nil	SC	Nil
II	30	7 Days	SC	Nil
III	30	7 Days	EC	Nil
IV	24	Nil	EC	Nil
V	06	7 Days	EC	K252a
VI	06	Nil	EC	K252a
VII	06	Nil	SC	TrkA Antisense
VIII	06	7 Days	EC	TrkA Antisense
IX	06	Nil	SC	TrkB Antisense
X	06	7 Days	EC	TrkB Antisense
XI	06	Nil	SC	U0216
XII	06	7 Days	SC	U0216
XIII	06	7 Days	EC	U0216
XIV	06	Nil	SC	Wortmannin
XV	06	7 Days	SC	Wortmannin
XVI	06	7 Days	EC	Wortmannin
XVII	06	Nil	SC	AR-A014418
XVIII	06	7 Days	SC	AR-A014418

### Housing Condition

Rats were randomly assigned to the enriched or the standard environmental condition. Enriched environment cages consisted of clear Plexiglas cages (35 inch ×20 inch ×25 inch) with two horizontal platform (20×15 inch) dividing the cage into three floors. On the ground floor, there was a plastic running wheel, nesting material and an assortment of differently colored and textured plastic toys (balls, tubes, boxes and bells) that were changed every 2 days. Steel ladders allowed rats to reach the upper floors, where they had access to food and water. Standard cages were clear Plexiglas laboratory cages (18×25×13 inch). Rats were kept in standard cage in groups of 3 each whereas in enriched cage they kept in group of 6 each. Enriched and standard cages were placed in a temperature-controlled room (22°C) with a light–dark 12∶12 cycle (light on 0700–1900 hrs). Food and water were given *ad libitum*. Rats were housed in each experimental condition for 7 days.

### Antisense and Inhibitors

To determine the role of neurotrophins, intracerebroventricular (ICV) injection of either vehicle (VEH; PBS, pH 7.4) or tyrosine kinase (Trk) inhibitor i.e., K252a was administered (250 µM, 5 µl) into the left hemisphere of adult rat brain.

The Trk gene silencing was performed *in vivo* by administering TrkA and TrkB antisense oligonucleotides before HH exposure to rats. The antisense TrkB sequence refers to the sequence from nucleotide 651 to 670 (5′ ACTGGCAGCTCGGGATGTCG-3′). The antisense nucleotide, complementary to that sequence was 5′- CGACATCCCGAGCTGCCAGT-3′. The antisense TrkA sequence (59- AACTGTTGTTGTGTCC-39) corresponds to nucleotides 623–638 of rat TrkA. A random oligonucleotide (59- GTAAATTGACCAGGAG-39) was used as a control. The oligonucleotides were dissolved in a buffer containing10 mM Tris-Cl, pH 7.2, and 1 mM EDTA to a final concentration of 200 mM. Antisense oligonucleotides and randomized controls have been designed and manufactured by Biognostik (Gottingen, Germany). Intracerebroventricular (ICV) injection of either vehicle (VEH; PBS, pH 7.4) or antisense was administered into the left hemisphere of adult rat's brain as described in supplementary information (Supplementary Information File S1). An ERK1/2 inhibitor, U0216; a PI3 kinase inhibitor, wortmannin and GSK3ß inhibitor, AR-A014418 were purchased from Sigma Aldrich (San Diago, CA). U0216 and Wortmannin were dissolved in PBS whereas AR-A014418 was dissolved in DMSO and administered before HH exposure at a concentration of 1nmol, 0.1nmol and 30 µmol respectively [18]. Rats were ICV injected with a 5 µl solution containing either VEH (1 µl of DMSO and 4 µl of PBS, pH 7.4) or inhibitor as stated above.

### Hypobaric hypoxia Simulation

Following probe trial the rats were divided into different groups as shown in Table 1. The hypoxic and hypoxic with enriched environment groups were exposed to a simulated altitude of 7600 m (25,000 ft) in a specially designed hypobaric chamber where altitude could be maintained by reducing the ambient barometric pressure. The exposure was for continuous 7 days with a 15 min interval each day during the exposure for replenishment of food and water and changing the cages of the animals. Fresh air was continuously flushed at a rate of 8 L/min to prevent accumulation of carbon dioxide within the chamber. The temperature and humidity in the chamber were maintained at 28±2°C and 60±3% respectively. The rate of ascent and descent was maintained at 300 m/min.

### Memory Assessment

Reference memory was assessed in Morris Water Maze [25]–[26] to investigate spatial learning and memory of rodents. Before HH exposure animals were trained for 8 days and probe trial was performed before and after HH exposure. Single task of memory test was performed after exposure to HH. Detailed protocol for training, probe trial and memory task are as follows.

Prior to exposure to hypobaric hypoxia rats were trained in a Morris water maze to study the effect of enriched environment on spatial reference memory acquisition. The maze comprised of a white circular pool of 180 cm diameter, filled with water (temperature around 24–25°C, depth 50 cm). The pool was conceptually divided into four equal quadrants having 4 points designated as starting positions (North, South, East or West). The pool had an escape platform submerged in water (2 cm below the water surface) which was camouflaged by mixing non toxic white paint to the water. The rats were painted black using a hair dye as the software detected the movements based on a phase contrast principle. The position of a black rat in the white maze was recorded by an overhead camera and computer assisted tracking system (Columbus instruments, USA).

#### (i) Training

The animals were divided into different groups and trained for 8^th^ days (sessions) and a probe trial was performed on the 9^th^ day. Each session consisted of four trials with a 15 min inter-trial interval. The platform position remained in the same location throughout the training period. A trial began when the rat was released into water facing the wall of the pool at one of the 4 starting positions that was chosen at random. The order of the starting position varied in every trial and any given sequence was not repeated in the next session. During the trial, the rat was allowed to locate the submerged platform for 60 s. If the animal failed to reach the platform it was gently guided to it and left on it for 10 s. The latency (in seconds) and pathlength (in cm) to find the platform was recorded in each trial and mean latency and pathlength for each session was calculated.

#### (ii) Probe Trial

Twenty four hours after the end of the last training on the eighth day, rats were subjected to probe trial, a task, which was designed to assess the consolidation and retrieval of reference memory. It consisted of a single trial wherein the rats were allowed to swim for 60 s, with the platform removed from its position. Here, the number of crossing over at the original platform position and the time (s) spent in the target quadrant were measured. Rats were found to spend maximum time in the target quadrant and the crossing over frequency averaged around 5 during the probe trail indicating consolidation of memory.

#### (iii) Memory test (testing for retention of learned task)

Rats in all the groups were immediately tested for memory retention following the stipulated period of 7 days exposure to hypobaric hypoxia for all groups. The rats were subjecting to a probe trial followed by a single trial of the task that was given during training for acquisition of spatial reference memory. The time spent and distance traveled to reach the platform, time spent in the target quadrant, and number of crossing over at the platform position was recorded during the probe trail.

### Sample Preparation

After exposure and memory assessment rats were deeply anesthetized with sodium pentobarbital (100 mg/kg, *i.p*.), perfused transcardially with chilled PBS and decapitated. The brain were dissected out and used for different experimental protocols accordingly.

### Neuronal death by Cresyl Violet Staining

After hypoxic exposure, rats were anesthetized and perfused with ice cold PBS, fixed with 4% paraformaldehyde, cryoprotected in 30% sucrose solution, sliced into 10 µm free floating sections and processed for Cresyl violet staining. Morphology of neurons in CA1 regions was studied. Briefly every sixth section from each individual was taken, dehydrated using gradient alcohol concentration, stained with cresyl violet for 3 mins and then rehydrated again. The sections were transferred to slides and mounted with permanent mounting media. Morphology of neurons in CA1 region was observed under light microscopy. Counting of pyknotic/dead cells was done using Stereo investigator (MBF Biosciences, USA).

### Neuronal degeneration

Neuronal degeneration was assessed histologically in each of the experimental groups by fluoro jade (FJ) B staining method as described previously [27]. Briefly, every sixth section from each individual was taken for assessment of neuronal degeneration in CA1 region in hippocampus. The sections were stained according to the protocol suggested by the manufacturers and sections were visualized at 480 nm excitation and 525 nm emission using a fluorescent microscope (OLYMPUS) with FITC filters. The total number of fluoro jade positive cells were scored in each of the regions and results were depicted in terms of percentage increase in fluoro jade positive cells taking average number of fluoro jade positive cells in normoxic group to be 100%.

### RNA isolation and PCR array

Total RNA was isolated from rat hippocampus using a Qiagen total RNA isolation kit according to the manufacturer's recommendations. Rat signal transduction pathway RT^2^ Profiler PCR Array and RT^2^ Real-Time SyBR Green/ROX PCR Mix were purchased from Super Array Bioscience (Frederick, MD). PCR was performed on ABI Step One Plus (Applied Biosystems), according to the manufacturer's instructions. Samples from all groups were compared. For data analysis, the ΔΔCt method was used with the aid of a Microsoft excel spreadsheet containing algorithms provided by the manufacturer. Fold-changes were then calculated and expressed as log-normalized ratios of values from all tissues.

### Immunoblotting

Samples from each group (50 µg) were loaded onto SDS-PAGE gels. Following electrophoresis gels were transferred by semi dry transblot (Biorad) to nitrocellulose membranes and probed against rabbit polyclonal AKT, pAKT, mouse monoclonal ERK, pERK and rabbit monoclonal GSK3ß, pGSK3ß, CREB and pCREB antibody (Sigma, St. Louis, Mo., USA) at a concentration 1∶1000, and further with respective secondary antibody labelled with horseradish-peroxidase at a concentration 1∶5000 (Santa Cruz, CA). The membranes were developed using the enhanced chemiluminescence light (ECL) (Sigma. USA) and then membrane was exposed to X-ray film for detection.

### DEVD-AMC cleavage assay

The Asp-Glu-Val-Asp-(7-amino-4-methylcoumarin) (DEVD-AMC) cleavage assay was performed as described previously (Jain et al.,2012). Acetyl-AMC (Calbiochem) was used to obtain a standard curve, and the enzyme activity was calculated as picomoles of AMC/mg of protein/min.

### Statistical Analysis

The data of 8 day acquisition trials in Morris Water Maze was averaged for each session of four trials. The performance during trials was analyzed using two-way Analysis of Variance (ANOVA) with trials as repetitive measures. In the probe trial task (single trial), at the end of 8 days training and again after exposure to hypoxia platform crossings, time spent in target quadrant in initial 10 s, was analyzed using one-way ANOVA. Similarly, mean of latencies and pathlength for reference memory testing after exposure to hypobaric hypoxia was analyzed in similar manner since a single trial was given to each animal during the task. The results of histology and all biochemical estimations are representations of 6 individual observations and statistical analysis for multiple comparisons was done using two-way ANOVA. Data is presented as mean ± SEM. Pair wise comparisons were used to evaluate the difference between different experimental groups. All analysis was followed by *post hoc* student's Newman's Keul's test, when necessary. Probability value ≤5% (p<0.05) was considered significant for all statistical analysis.

## Results

### Enriched Environment (EE) improves spatial memory during hypobaric hypoxia

Morris Water Maze task training for 8 days leads to progressive improvement in the ability of rats to explore the hidden platform in the target quadrant (Fig. 1). Exposure to HH for seven days significantly (p<0.001) increases the pathlength (Fig. 1A) and latency (Fig. 1B) of rats. The group kept in EE housing during HH showed significant (p<0.001) decrease the pathlength and latency of rats when compared to group exposed to HH without EE.

**Figure 1:** Behavior changes was studied using Morris Water Maze test and representative tack sheet showing memory test of Control (I), Hypoxia (II), Enriched environment with Hypoxia (III) and Enriched environment without hypoxia (IV) exposure. Latency (A) and Pathlength (B) were increased on HH exposure whereas EE revert back these effects to normal. In contrast HH leads to lessen the number of platform crossing (C) and time spent in target quadrant (D) and EE again showed promising effect by increasing their value. Data represents Mean ± SEM. “*” and “#” represents p<0.001 when compared to control and hypoxic group whereas “**” represents p<0.05 when compared to hypoxic group.

Probe trial data of rats exposed to HH shows significant decrease in inclination towards the target quadrant as evident from number of platform crossing (Fig. 1C) and time spent in target quadrant (Fig. 1D) when compared to control group. Conversely the group housed in EE cage during HH and normoxia spent maximum time in target quadrant with increased number of platform crossing.

### Enriched environment provides neuroprotection against hypobaric hypoxia mediated cell death

Neuronal degeneration as observed by Fluoro jade B staining increased on exposure to HH. Increased number of Fluoro jade B positive cells (84.2±4) (Fig. 2) was observed in the CA1 region of hippocampus in group exposed to HH when compared to the control (34.1±3.2). Providing EE during exposure to HH on the other hand significantly decreased (57.5±4.9) the number of Fluoro jade B positive cells. The neuronal degeneration in enriched environment groups was considerably lower than animals subjected to similar duration of exposure in standard environment.

**Figure 2:** Fluoro Jade (FJ) and Cresyl violet staining, was assessed to study neurodegeneration and cell morphology. It was observed that Hypobaric hypoxia leads to neurodegeneration and cell pyknosis as evident from increased number of FJ positive cells and pyknotic cells whereas enriched environment decreases number when compared to hypobaric hypoxia alone group. Data represents Mean ± SEM. “*” and “**” represents p<0.001 when compared to control and hypoxic group.

Cell morphology was also studied using cresyl violet staining. Results showed that exposure to HH leads to cell pyknosis and shrinkage in CA1 region of hippocampus which confirms previous findings [28]. Similar to above finding, cresyl violet staining also showed that EE prevents hypobaric hypoxia induced altered cell morphology as number of pyknotic cells were decreased on providing EE during exposure to HH (Fig. 2).

### Enriched environment prevents memory impairment through Trk signaling

To further assess the role of neurotrophins mediated Trk activation in EE mediated memory improvement during HH, Trk receptor was inhibited with an antagonist, K252a. Results showed that EE fails to ameliorate HH mediated memory impairment in presence of Trk antagonist i.e. K252a (Fig. 3) as evident from increased path-length (Fig. 3A), latency (Fig. 3B), decreased time spent in target quadrant (Fig. 3C) and number of platform crossing (Fig. 3D). This shows that Trk signaling plays an important role in EE mediated amelioration of spatial memory impairment.

**Figure 3:** Effect of Trk antagonist on Behavior was studied using Morris Water Maze test and representative tack sheet showing memory test of Normoxia (I), Hypoxia (II), Enriched environment + Hypoxia (III) and Enriched environment + hypoxia + K252a (IV) exposure. Inhibition of TrkB with K252a nullifies the protective effect of Enriched environment on hypobaric hypoxia induced memory impairment as evident from increased pathlength (A) and latency (B) and decreased No. of platform crossing (C) and time spent in target quadrant (D). Data represents Mean ± SEM. “*” and “#” represents p<0.001 when compared to control and hypoxic group whereas “**” represents p<0.05 when compared to hypoxic group.

### Knockdown of TrkB expression impairs EE mediated neuroprotection

Trk receptor is involved in BDNF and NGF mediated signaling and has its own importance in cell biochemistry [24]. In present study the role of specific neurotrophin (BDNF or NGF) was studied using gene silencing method. For this TrK gene silencing was performed *in vivo* by using antisenses for TrkA and TrKB receptors. Results showed that administration of antisense oligonucleotides for TrkA and TrkB during exposure to HH in EE significantly decreased their expression as shown by immunoblotting (Figure S1 in File S1) Caspase3 activity was assessed to evaluate apoptotic cell death in hippocampus after antisense administration. Findings of present study showed that silencing TrkB expression with antisense significantly increased apoptotic cell death even in presence of EE as evident from increased caspase3 activity whereas silencing TrkA expression has little or insignificant effect on caspase3 activity (Fig 4A).

**Figure 4:** Role of neurotrophins was assessed using gene silencing technique for TrkA and TrkB receptors. Results showed that knockdown of TrkB significantly increased caspase3 activity even in presence of enriched environment whereas blocking of TrkA has diminutive effect on caspase3 activity in comparison to TrkB inhibition. To further explore the signaling cascade, ERK and PI3K pathway was blocked with U0216 and Wortmannin respectively and it has been observed that inhibition of PI3K pathway significantly increases caspase3 activity (B) whereas inhibiting ERK pathway have no significant effect in group exposed to hypobaric hypoxia in enriched cage (C). Data represents Mean ± SEM. In “*” and “#” represents p<0.001 when compared to control and hypoxic group while “?”represents p<0.05 when compared to control group.

### Activation of PI3K/AKT pathways is essential for BDNF mediated neuroprotection

BDNF mediated TrkB activation is well known for neuronal survival *via* various signaling pathways under different conditions. In present study, results of PCR array showed fold changes in survival genes like Bcl2, Ccnd1, Fn1, Jun, Mmp7, Myc, Pten in group placed in EE with concurrent exposure to HH (Table S1 in File S1). These genes are related to both PI3K and ERK pathways which may play a role in EE mediated neuroprotection. Further validation with western blot for protein level showed that enriched environment mediated BDNF up-regulation activates both pathways via phosphorylation of ERK1/2 and AKT with greater percent increase in pAKT than pERK over baseline (Figure S2 in File S1). Despite the BDNF stimulated increase in pERK and pAKT, no changes were observed in total AKT and ERK levels.

To address possible role of ERK pathway in EE mediated neuroprotection, pathway was blocked using inhibitor U0216, that prevents ERK phosphorylation and hence its activation. Results showed that administering U0216 markedly inhibit the increase in pERK1/2 without affecting the EE mediated pAKT increase. Administration of U0216 during HH has no significant effect on caspase-3 like activity in group housed in EE in comparison to vehicle (Fig. 4C). These results suggest that BDNF mediated activation of ERK pathways does not appear to play a major role in EE mediated neuroprotection.

Further role of PI3K pathway in EE mediated neuroprotection was also assessed by blocking BDNF stimulated PI3K activation without inhibiting the pERK increase. Wortmannin was used to inhibit PI3K/AKT pathway by blocking AKT phoshorylation. Results showed that blocking PI3K/AKT pathway with wortmannin markedly increase the caspase-3 activity in group housed in enriched environment when compared to vehicle (Fig. 4B). These findings put forward major contribution of PI3K pathway in EE mediated neuroprotection *via* BDNF stimulation.

### Role of GSK-3β in EE mediated neuroprotection

Role of Glycogen Synthase Kinase 3 Beta (GSK-3β) in EE mediated neuroprotection was also investigated and it was observed that HH exposure causes GSK-3β activation as evident from decreased level of GSK-3β phosphorylation whereas concurrent exposure to EE prevents this activation (Fig. 5A). Role of TrkB receptor on GSK-3β inactivation was also studied and it was found that inhibiting TrkB expression reduced GSK-3β phosphorylation (Figure S3 in File S1). Moreover the inhibition of PI3K/AKT with Wortamannin significantly increases the activation of GSK-3β (decreases GSK-3β phosphorylation), even in presence of EE whereas on blocking ERK pathway with U0216, no significant change in activation of GSK-3β was observed.

**Figure 5:** Downstream cascade was further explored and it was shown that hypobaric hypoxia reduces GSK3ß phosphorylation (A) and hence its inactivation whereas enriched environment significantly ameliorate this effect. In presence of PI3K inhibitor (Wortmannin) enriched environment have little effect on GSK3ß phosphorylation. Inhibition of ERK pathway with U0216 showed no significant effect on GSK3ß phosphorylation. Moreover hypobaric hypoxia also decreases the CREB phosphorylation (B) whereas exposing them with enriched environment normalizes this decreased level of CREB phosphorylation. Similarly inhibition of GSK3ß with AR-A014418 elevates the CREB phosphorylation equivalent to group exposed to enriched environment during hypobaric hypoxia. Data represents Mean ± SEM. In “*” and “#” represents p<0.001 when compared to control and hypoxic group while “?”represents p<0.05 when compared to control group.

### GSK-3β inhibition mediate CREB activation

Further it was postulated that EE mediated GSK-3β inhibition may activate cAMP response element-binding (CREB). Findings from present study showed that HH decreases phosphorylation of CREB by upto 2 fold (50%) in comparison to control; whereas on concurrent exposure with EE the phosphorylation of CREB reverts to normal level. Additionally, inhibiting GSK-3β activity with inhibitor, ARA014418 during HH also restored the phospho-CREB level to normal (Fig. 5B). No changes were observed in total CREB level in all the groups.

## Discussion

Chronic exposure to HH leads to memory impairment in rats [28] which may attribute to various factors including glutamate excitotoxicity, alteration in cellular biochemistry, depletion of growth factors etc. which may lead to cell death. It was reported that hippocampus is found to be more prone to HH in comparison to other brain regions [29]. Distinctly hippocampus is known to be activated by social interactions [30], exposure to novel environments [31] and the spatial rearrangement of familiar objects of the environment [32]. Previously, we have reported that EE provides neuroprotection against HH mediated neurodegeneration through antioxidant independent signaling [24]. An important upshot is to understand the signaling mechanism involved in EE mediated neuroprotective effects in models of relevant diseases of the nervous system. Present study was designed to elucidate the effect of EE on HH induced memory impairment and also to explore the possible role of neurotrophins mediated signaling in EE mediated neuroprotection. Findings of the present study confirms the EE mediated amelioration of HH induced memory impairment and also explored the role of BDNF mediated PI3K activation which further leads to GSK3β inhibition coupled with CREB up-regulation and prevents neurodegeneration.

The reference as well as working memory gets impaired on chronic exposure to HH [33]. The results of the present study showed that EE improves spatial memory in rats exposed to chronic HH (7 days) as evident from decreased latency and pathlength and significant increase in time spent in target quadrant. Similarly, the number of platform crossing also increased in Morris Water Maze task. The results of the present work is found to be in accordance with several other studies which reported that EE prevents chronic stress-induced spatial learning and memory deficits [34], whereas study of Tauber et al observed that EE fails to improve spatial memory in model of pneumococcal meningitis [35]. The reason behind such contradiction may be due to different time points of providing enriched environment as well as severity of stress.

The EE is known to provide neuroprotection against many neurodegenerative disorders like focal cerebral ischemia, hypoxia-ischemia, depression, Huntington's disease and Alzheimer's disease [36]–[37]. Hippocampus has been reported to be more prone to HH in comparison to other brain regions and maximum damage was found in CA1 region of hippocampus [28], [38]. Finding of present study also indicated that chronic exposure to HH exposure leads to neurodegeneration as evident from increased number of Fluoro Jade positive cells in CA1 region of rat hippocampus. Whereas exposing them with EE during HH prevented neurodegeneration and decreased the number of Fluoro Jade positive cells. Similar results were found in a study of Hu et al., where EE attenuates neuropathology and synaptic plasticity in Alzheimer's disease [37]. Additionally EE also showed promising effect on altered cell morphology by plummeting HH mediated cell pyknosis. These multifaceted morphological effects of EE may connect to the significant involvement of a sensory-motor circuit engaged in the guidance of voluntary action and in motor learning activated by EE stimulation.

The mammalian neurotrophins, nerve growth factor (NGF), brain derived neurotrophic factor (BDNF), neurotrophin-3 (NT-3) and neurotrophin 4/5 (NT-4/5), all have been shown to play an essential role in neuronal viability and differentiation, as well as synaptic plasticity in various brain regions relevant to learning and memory [39]. Two types of receptors mediate neurotrophins action: high affinity membrane-bound tyrosine kinase receptors (Trk) and a low affinity pan-neurotrophin receptor (p75). Specific Trk receptors have preferential affinities for one or more of the NTs: TrkA for NGF, TrkB for BDNF and NT-4/5, and TrkC for NT-3. BDNF is one member providing a target derived signal for the establishment of neuronal connections during development, as well as continuing to modify these networks long after their establishment [40]. In present study, tyrosine kinase (Trk) receptor inhibition with K252a nullifies the beneficial effect of EE on spatial memory as evident from Morris water maze task. Henceforth, it provides strong evidence for involvement of Trk signaling in EE mediated amelioration of HH induced memory impairment. Previously it has been shown that blocking Trk with K252a increases caspase3 expression in CA1 region of hippomcapus [24]. Similar findings were observed in a study of Nitta et al which showed that exogenous administration of neurotrophins attenuated corticosterone induced neural death but in presence of Trk inhibitor (K252a) the effect was abolished [41]. Furthermore, result from present study also demonstrated that of all the Trk receptors, knocking down of TrkB receptor during HH using antisense technique significantly increases apoptosis even in presence of enriched environment as evident from increased caspase3 activity whereas knockdown of TrkA receptor has no significant effect. This indicates that the contribution of BDNF mediated TrkB activation is a necessary event in EE mediated neuroprotection against chronic HH. Similar type of result was also reported by Faherty et al, which showed that the EE provide neuroprotection against Parkinson disease through up-regulation of BDNF [9]. Whereas some studies also showed that EE fails to provide protection and reveres reduced level of BDNF following axotomy and hypoxia-ischemia [42]–[43]. These contradictory results may be due to variation in stress condition because of different durations of exposure to EE used according to planned studies.

The BDNF mediated TrkB activation known to provide neuroprotection through alteration of various pathways but mainly two pathways shows utmost contribution (ERK and PI3K pathway). The PCR array results from present study showed significant fold changes of expression of the genes involved in survival pathway in EE condition and major difference was found in genes (Bcl2, Ccnd1, Fn1, Jun, Mmp 7, Myc, Pten) involved in PI3K and ERK pathway. Based on these observations, it can be postulated that EE mediated neuroprotection requires activation of both ERK and PI3K pathway. Further both pathways were inhibited alternately with the help of respective blockers *i.e*. U0216 for ERK and Wortmannin for PI3K and it was observed that blocking of PI3K pathway nullifies the effect of EE mediated neuroprotection against HH significantly, whereas ERK has no significant contribution in EE mediated neuroprotection by BDNF stimulation. Our findings are found to be supporting various other studies which showed that BDNF provide neuroprotection against brain pathology *via* activation of PI3K/AKT pathway [43]. Whereas some studies also showed that BDNF stimulates ERK pathway against hypoxia-ischemia [18]. The study of Hetman et al. emphasizes that the stressful stimulus can determine which pathway is dominant even within the same cell type [17]. It was found that in response to serum deprivation, BDNF mediated survival of cultured cortical neurons *via* the PI3-kinase pathway. In contrast, when the same cells were treated with campothecin, a DNA synthesis inhibitor, BDNF mediated protection *via* ERK pathway [17].

The GSK-3β as a pro-apoptotic factor is important for neuronal apoptosis cascade and also reported to be crucial for PI3Kmediated neuronal survival [19]. In its active form GSK-3β enhance apoptosis whereas on phorphorylation GSK-3β become inactive and unable to trigger apoptotic pathway. Present study showed that EE inactivates GSK-3β by increasing its phosphorylation and hence prevents apoptosis during HH through TrkB activation (Figure S3 in File S1). Also, inhibiting PI3K/AKT pathway with Wortmannin prevented EE mediated GSK-3β phosphorylation and hence caused inactivation, whereas inhibiting ERK pathway with U0216 fails to generate same effects. This implies that GSK-3β phosphorylation mediated by EE evoked BDNF which is completely dependent on the PI3K/AKT axis and seems to be unaffected by ERK inhibition. Some findings showed that GSK-3 phosphorylation and neuroprotection becomes MAPK dependent only when the PI3K/AKT axis is impaired. Therefore, it points out that the ERK proteins acts as an alternative for GSK-3β phosphorylation and hence inactivation [44].

CREB is a key transcription factor involved in several critical functions of the brain including learning, neuronal plasticity and cell survival [45]. CREB has been shown to be the key mediator for BDNF-mediated cell survival as studies showed that silencing the transcriptional activity of CREB impaired BDNF protection [46]. CREB can be activated by various kinases including ERK, AKT and GSK-3β [47]. Our finding showed that HH decreases CREB phosphorylation when compared to normoxia. However providing EE during HH restored the CREB phosphorylation to its normal level. Similarly, inhibiting GSK-3β activity with AR-A014418 also prevented HH induced decrease in CREB phosphorylation. Bearing in mind that EE through BDNF inhibit HH mediated GSK-3β activation, we put forward that EE may increase CREB activity through BDNF mediated inhibition of GSK-3β activity. This activated CREB may further regulate the transcription of several genes involved in cells survival mechanism.

The present study concluded that EE prevents spatial memory impairment during HH. Further these beneficial effects of EE are induced *via* BDNF stimulated PI3K activation which inhibits GSK-3β activation. Further GSK-3β inactivation through its phosphorylation directly inhibits apoptosis. Moreover inactivation of GSK-3β also leads to CREB phosphorylation which may regulates survival machinery of cells results in neuroprotection against HH (Fig. 6). Therefore BDNF and respective downstream molecules of PI3K pathway may prove to be good therapeutic targets against neurological disorders that cause memory impairment.

**Figure 6:** Schematic diagram of signaling events in enriched environment mediated neuroprotection during hypobaric hypoxia.

## Supporting Information

File S1 Knockdown of TrkA and TrkB with antisense techniques shows promising inhibition of expression of their respective receptors as shown in **Figure S1**. **Figure S2** describes TrkB mediated activation of ERK and PI3K pathways. Western blot analysis showed that inhibition of ERK pathway with U0216 and PI3K pathway with Wortmannin decreased the expression of pERK (A) and pAKT (B) respectively without altering their basal level. Interestingly it has been observed that knocking down the TrkB receptor fails to phosphorylate GSK3b and hence inactivation even in presence of enriched environment as shown in **Figure S3**. This shows that in present case BDNF mediated TrkB activation is necessary event for GSK3b inactivation. Data represents Mean ± SEM. “*” and “**#**” represents p<0.001 when compared to control and hypoxic group respectively whereas “**” represents p<0.05 when compared to control group.
(DOC)
